# The OMOP common data model in Australian primary care data: Building a quality research ready harmonised dataset

**DOI:** 10.1371/journal.pone.0301557

**Published:** 2024-04-18

**Authors:** Roger Ward, Christine Mary Hallinan, David Ormiston-Smith, Christine Chidgey, Dougie Boyle

**Affiliations:** Health & Biomedical Research Information Technology Unit (HaBIC R2), Department of General Practice and Primary Care, Faculty of Medicine, Dentistry & Health Sciences, The University of Melbourne, Parkville, Victoria, Australia; Kyung Hee University School of Medicine, REPUBLIC OF KOREA

## Abstract

**Background:**

The use of routinely collected health data for secondary research purposes is increasingly recognised as a methodology that advances medical research, improves patient outcomes, and guides policy. This secondary data, as found in electronic medical records (EMRs), can be optimised through conversion into a uniform data structure to enable analysis alongside other comparable health metric datasets. This can be achieved with the Observational Medical Outcomes Partnership Common Data Model (OMOP-CDM), which employs a standardised vocabulary to facilitate systematic analysis across various observational databases. The concept behind the OMOP-CDM is the conversion of data into a common format through the harmonisation of terminologies, vocabularies, and coding schemes within a unique repository. The OMOP model enhances research capacity through the development of shared analytic and prediction techniques; pharmacovigilance for the active surveillance of drug safety; and ‘validation’ analyses across multiple institutions across Australia, the United States, Europe, and the Asia Pacific. In this research, we aim to investigate the use of the open-source OMOP-CDM in the PATRON primary care data repository.

**Methods:**

We used standard structured query language (SQL) to construct, extract, transform, and load scripts to convert the data to the OMOP-CDM. The process of mapping distinct free-text terms extracted from various EMRs presented a substantial challenge, as many terms could not be automatically matched to standard vocabularies through direct text comparison. This resulted in a number of terms that required manual assignment. To address this issue, we implemented a strategy where our clinical mappers were instructed to focus only on terms that appeared with sufficient frequency. We established a specific threshold value for each domain, ensuring that more than 95% of all records were linked to an approved vocabulary like SNOMED once appropriate mapping was completed. To assess the data quality of the resultant OMOP dataset we utilised the OHDSI Data Quality Dashboard (DQD) to evaluate the plausibility, conformity, and comprehensiveness of the data in the PATRON repository according to the Kahn framework.

**Results:**

Across three primary care EMR systems we converted data on 2.03 million active patients to version 5.4 of the OMOP common data model. The DQD assessment involved a total of 3,570 individual evaluations. Each evaluation compared the outcome against a predefined threshold. A ’FAIL’ occurred when the percentage of non-compliant rows exceeded the specified threshold value. In this assessment of the primary care OMOP database described here, we achieved an overall pass rate of 97%.

**Conclusion:**

The OMOP CDM’s widespread international use, support, and training provides a well-established pathway for data standardisation in collaborative research. Its compatibility allows the sharing of analysis packages across local and international research groups, which facilitates rapid and reproducible data comparisons. A suite of open-source tools, including the OHDSI Data Quality Dashboard (Version 1.4.1), supports the model. Its simplicity and standards-based approach facilitates adoption and integration into existing data processes.

## Introduction

The use of routinely collected health data for secondary research purposes is increasingly recognised as a methodology that advances medical research, improves patient outcomes, and guides policy [1–4]. This secondary data, as found in electronic medical records (EMRs), can be optimised through conversion into a uniform data structure to enable analysis alongside other comparable health metric datasets [4–6]. This can be achieved using the Observational Medical Outcomes Partnership Common Data Model (OMOP-CDM), which employs a standardised vocabulary to facilitate systematic analysis across various observational databases. The OMOP-CDM is a data schema that uses a standardised vocabulary for the systematic analysis of multiple distinct observational repositories (databases) [7]. The concept behind the OMOP-CDM, is the conversion of data into a common format through the harmonisation of terminologies, vocabularies, and coding schemes within a unique repository (Fig 1) [7].

**Fig 1:** OMOP common data model architecture [7, 12].

The primary purpose of an EMR is to record information related to patient care as it naturally occurs in the clinical setting [8]. The use of this data in medical research is a secondary, albeit useful function, as it provides the opportunity to establish ‘real world’ evidence on patient outcomes, healthcare quality, comparative effectiveness, and health system policy [9]. Yet, the quality of data recorded in an EMR varies in its completeness, conformance, plausibility, and currency, hence it is imperative that a measure of its quality is ascertained to determine if is suitable for research purposes. Kahn et. al. [10] established a comprehensive set of quality checks that have since become the widely adopted ’de facto’ standard across the globe. We used these standards to ascertain data quality in this research.

The OMOP model enhances independent institutional research capacity through the development of: shared advanced analytic and prediction techniques; pharmacovigilance for the active surveillance of drug safety; and ‘validation’ analyses across multiple institutions across Australia, the United States, Europe and the Asia Pacific [7]. In this research we aim to investigate the use of the open-source OMOP-CDM in the PATRON primary care data repository [11].

## Methods

### Data warehouse

The dataset was sourced from a data warehouse Primary Care Audit, Teaching and Research Open Network Program (PATRON) curated by the University of Melbourne [11]. The database collects de-identified EMR data from 129 Australian general practices, chiefly in Victoria. The repository comprises over 700 consenting general practitioners (GPs) who work in Australian general practices that use Best Practice™, Medical Director™, and ZedMed™ proprietary EMR systems (Table 1).

**Table 1:** Types of EMR systems studied.

EMR	URL	General Practice n (%)
Medical Director (MD)	https://www.medicaldirector.com	52/129 (40%)
Best Practice (BP)	https://bpsoftware.net	65/129 (50%)
Zedmed	https://www.zedmed.com.au	12/129 (10%)

EMR data are extracted from these systems using the data extraction tool GRHANITE™ [13], and the data is then sent via encrypted transmission into the repository. The GRHANITE™ tool de-identifies each patient by replacing the patients name with a unique patient identifier that links the patient to the individual visit data in each patient table [13]. Identifiers including patient address, date of birth, Medicare number (i.e., health insurance number/healthcare identifier), general practitioner, and staff member details are either removed or deidentified prior to extraction to the data repository.

Each EMR system held in the PATRON repository has a data structure that is unique. Hence, to facilitate use of the whole database, the data from each system are harmonised to provide consistency. For instance, to provide a standardised version to the database, all data pertaining to ‘patient history’ from each EMR are merged into a single table, and likewise information relating to ‘medications prescribed’ are also merged into a table. Whilst data standardisation provides a single unified view to simplify researcher use, no data is lost in this harmonisation process (Fig 2).

**Fig 2:** EMR harmonisation process.

### Mapping process

Primary care EMR systems incorporate both free text terms and proprietary coding, which is uniquely specified by each individual EMR vendor. Therefore, one of the challenging aspects of extracting meaningful data is mapping the free text data to numerical codes in vocabularies such as the Systematized Nomenclature of Medicine Clinical Terms (SNOMED) and RxNorm (United States, medication terminology). It is important to note SNOMED is considered the ‘standard terminology’ for conditions in the OMOP CDM, and likewise, RxNorm is the ‘standard’ for medications. An additional advantage of employing these vocabularies for the preparation of data for OMOP compatibility, is that the mapping process results in a repository that conforms to international standards.

The mapping process was facilitated through the utilisation of a tool called USAGI, developed by the multi-stakeholder international collaborative body, Observational Health Data Sciences and Informatics (OHDSI) [7]. The USAGI tool is crafted with the purpose of transforming text terms extracted from the data warehouse into standardised SNOMED and RxNorm terms. Despite its utility, USAGI still relies on manual input from data mappers who possess specialised domain knowledge. This expertise is essential for ensuring the accuracy of the mapping process, as it enables a deep understanding of the clinical expertise within the field of medicine, guaranteeing precise representation of medical conditions and treatments. In our approach, we enlisted the expertise of three final-year medical students, these students independently conducted data mappings, where pairwise comparisons of their mappings were assessed for concordance using Excel. There was a ninety percent agreement in the student mappings, clinical insights from a physician were sought to resolve discrepancies.

The volume of distinct free text terms from each unique EMR within the PATRON data repository presented challenges. For example, there were 96,000 distinct medication terms, consisting of some combination of a drug’s brand name, generic name, form, strength, and packet size. Only a small fraction, less than five percent, could be automatically linked to the standard RxNorm concept through direct text matching. This left a substantial number of terms requiring manual assignment. To manage this, our mappers were instructed to map all terms that occurred with sufficient frequency.

For each domain, we set specific threshold values to ensure that over ninety-five percent of all records were associated with an appropriately mapped SNOMED or RxNorm concept. As a result, terms occurring 200 times, or more were mapped. A similar approach was taken for fields other than medications. For example, in the ’reason for visit’ table, only conditions that occurred 50 or more times were mapped.

There was no direct match of a ‘conditions’ table in the EMR to the ‘conditions occurrence’ table in the OMOP-CDM. Unlike the OMOP-CDM, which integrates pertinent SNOMED terms into a unified ’condition occurrence’ table to depict a patient’s condition, the EMR uses separate ’reason for visit’ and ’history’ tables to store information about a patient’s current condition, past medical history, and clinical observations.

If an entry in the EMR was accompanied with a date, we considered it a current condition and recorded it as a ‘condition occurrence’ in the OMOP table. Conversely, when a condition did not have an associated date, we considered it as a past observation and therefore recorded it as an ‘observation’ in the OMOP-CDM.

### Extract Transform and Load (ETL) Structured Query Language (SQL) scripts

We used mapping tables, constructed from the mappings generated by the mapping team, to facilitate the transformation of EMR data into the OMOP-CDM during the Extract, Transform, and Load (ETL) process.

ETL incorporates the process of retrieving data from a source system, converting it into the format specified by the OMOP model, and then inserting it into the OMOP-CDM database. This transformation is achieved through the use of SQL scripts, which are sets of instructions designed to manage and modify data within the database.

### Removal of inactive patients

The Royal Australian College of General Practitioners (RACGP) employs ‘active patients’ as the specific group or denominator for the purpose of reporting clinical indicator measures [14]. This ensures clinical indicator assessments and reports refer only to patients who care classified as ‘active’ or ‘current’ within their practice. As per RACGP definition of an ‘active patient’, an inactive patient’ is defined a someone who has not attended a practice at least three times in the past two years [14]. Initially, this ‘inactive’ definition was applied to the dataset and the inactive patient records were excluded from the analysis. However, we found adherence to this definition resulted in the exclusion of new patients, with only 1 visit, so we also included patients with at least one visit over the last 2 years into the data set.

### Data analysis

Once the primary care data was converted into an OMOP compliant format it was securely connected to the ATLAS application for data visualisation and analysis purposes.

### Data governance

For research using the OMOP-CDM, a data governance framework has been developed building on the existing comprehensive framework implemented for primary care repository (Fig 3). This framework encompasses various topics including consent, privacy, and risk management [12, 15]. All governance procedures employed in our analysis were underpinned by the principal of *beneficence* ‘to do no harm’ [16].

**Fig 3:** The governance model.

### Consent

Medical practices provided consent for their practice data to be accessed for research purposes via the primary care repository. Practices are also informed they can change their consent options or withdraw at any time, without prejudice. Regarding individual patient consent for the secondary use of their EMR data, a waiver of consent is applied. A ’waiver of consent’ is often granted under the premise of ’easy rescue,’ where the perceived benefits of data access are deemed substantial, and the potential harm from the risk of privacy loss is considered minimal [17]. Practices inform patients their data is used for research using various communication strategies (i.e., on practice websites and practice posters), they are also informed they can withdraw consent at any point.

### Patient privacy

The GRHANITE™ data extraction tool de-identifies patient data in the practice before it is sent to our primary care repository. At no point is identifying data present within PATRON.

### Risk management

We conducted a structured risk assessment of the entire process considering privacy, organisational, and technical risks (Table 2).

**Table 2:** OMOP primary database assessment of risk.

Identified Risks	Risk Controls	Risk Rating
An authorised user discloses data to a third party.	Development of an access control policy based on researcher compliance with ethical, legal, and regulatory obligations related to privacy, data management, and data security.	Low
	Access to data on the OMOP platform is not provided if ethics approval is not verified.	
Unauthorised Intrusion by IT system ‘hackers	Application of strong passwords and multifactor authentication.	Low
	System not connected to public network.	
	Immediate notification of all data privacy/security breaches to the University of Melbourne to mitigate cybersecurity attack.	
Individual data is identified in the dataset.	Unique hash ID identifiers cannot be accessed via OMOP-ATLAS interface.	Low
	Data aggregation is possible at any level so that only required data is exported.	
Data accessible to researchers outside approved institutions	Currently only authorised researchers are permitted to analyse OMOP data operate OMOP within the University of Melbourne environment.	Low
Data changes or becomes corrupt.	Version control where the most recent database is always held as back up.	Low
	System identification of data extract failures or omissions for immediate notification to engineers.	
Researcher uses data for purposes beyond their ethics permissions.	User requires ethical approval and training to access the data.	Medium
	User accepts professional responsibility to adhere to boundaries of permissions.	
	Users restricted by OMOP- database access permissions.	
	External users are restricted by contractual agreement regarding their use of the data. Internal University staff are restricted by employment conditions and Memorandum of Understanding regarding their use of the data.	

## Results

### Data

The PATRON repository contains data for circa 5.6 million patients, which we harmonised. The results were harmonised and converted to version 5.4 of the OMOP Common Data Model (Table 3).

**Table 3:** Data in the data repository and the resultant OMOP CDM after conversion.

Data Metric	Number	Characteristics
Number of patients	5,564,425	Total database pool (Patients table)
Number of active patients	2,029,961	Number of patients in database with at least 3 visits within any 2 year-period, or that have at least one visit from the last 2 years.
Number of active patients with record of gender	2,023,161	A patient’s gender is one of:
		Female (1,086,934, 53.7%)
		Male (924,140, 45.7%)
		Not Recorded (11,526, 0.6%)
		Other (494, <0.1%)
		Unknown (67, <0.1%)
Number of clinical tables	15 clinical tables, but no data recorded in NOTE, NOTE_NLP, VISIT_DETAIL	As per OHDSI CDM definition there are 15 clinical tables, 3 health system tables, 2 health economics tables, 5 derived tables and 2 metadata tables.
		An additional 12 vocabulary tables exist that are prepopulated in the CDM.
Source database size	1.38 Terra Bytes (TB)	Original SNAPSHOT 1,383,296 MB
		Relevant Views rendered as tables (OMOP_SNAPSHOT_INSTANCE):
		778,193 Mega Bytes (MB)
CDM database size	0.37 TB	OMOP_CDM 368,512 MB

### Mappings

As described above, we mapped a term from the EMR if it exceeded a specified frequency threshold. This threshold level was established individually for each table (Table 4).

**Table 4:** EMR tables and related tables in the OMOP CDM.

EMR Source Table	Frequency threshold	CDM Output Table
Reason for Visit	50+	CONDITION_OCCURRENCE (if a condition with a date)
		OBSERVATION (if an observation)
History	100+	CONDITION_OCCURRENCE (if recorded with a date)
		OBSERVATION, MEASUREMENT (where no date)
		PROCEDURE_OCCURRENCE (if data is a procedure)
		DEVICE_EXPOSURE* (if data is a device)
Medications	200+	DRUG_EXPOSURE* (if data is a drug)
		DEVICE_EXPOSURE (if data is a device)
Immunisations	5+	PROCEDURE_OCCURRENCE
		DRUG_EXPOSURE*
Allergic reactions	20+	Stored as observation in
		OBSERVATION table
Tests	300+	DEVICE_EXPOSURE*
		MEASUREMENT
		PROCEDURE_OCCURRENCE data

*DEVICE EXPOSURE entity represents exposures to medical devices. Medical devices for medications are instruments, apparatuses, machines, implants, or similar items used in the pharmaceutical treatment of disease or injury.

### Medications occurrence

To illustrate the frequency-based approach for mapping, Table 5 shows the numbers that appear in the medications table in the EMR’s.

**Table 5:** Medication table mappings.

Category	Number of unique terms	Term Coverage
Distinct drug terms in EMR, post-cleaning	96,212	100%
Terms with incidence 200+	10,051	96.8% (49,460,151 out of 51,071,733 drug exposure records total)
Mapped terms (includes terms with incidence < 200, including mappings inherited from OMOP conversions performed by University of NSW, or those found via direct text match)	30,010	96.3% (49,193,190 out of 51,071,733 drug exposure records total)
Unmapped terms (includes terms with incidence > 200 where the term is insufficiently precise e.g., yearly influenza vaccinations, which often do not specify the specific formulation and thus cannot be mapped to the appropriate RxNorm concept)	66,202	3.7% (1,878,543 out of 51,071,733 drug exposure records total)

### Data quality

This data quality DQD assessment comprised a total of 3,570 individual evaluations. Each evaluation compared the outcome against a predefined threshold. A ’FAIL’ occurred when the percentage of non-compliant rows exceeded the specified threshold value. In this assessment of the primary care OMOP database described here, we achieved an overall pass rate of 97 percent (Table 6).

**Table 6:** OMOP results as of 20/10/22.

Quality indicators	Verification				Validation				Total			
	Pass (n)	Fail (n)	Total (n)	Pass (%)	Pass (n)	Fail (n)	Total (n)	Pass (%)	Pass (n)	Fail (n)	Total (n)	Pass (%)
Plausibility	1982	53	2035	97%	285	2	287	99%	2267	55	2322	98%
Conformance	746	30	776	96%	157	0	157	100%	903	30	933	97%
Completeness	289	14	303	95%	6	6	12	50%	50	295	20	94%
Total	3017	97	3114	97%	448	8	456	98%	3465	105	3570	97%

## Discussion

### The project

In our study, we conducted a comprehensive investigation into the implementation of the open-source OMOP-CDM in a primary care data repository. Utilising a substantial primary care dataset, we underscored the potential and wide-ranging implications of integrating the OMOP-CDM into real-world primary care settings. Additionally, we ascertained that adhering to the OHDSI-recommended conversion processes proved to be both practical and adaptable for achieving our research objectives.

The OMOP common data model proved to be a logical extension of our existing data warehouse. Once the tables and ETL scripts were established it proved to be simple to re-run the process every time we ran a new data extraction. As the CDM is primarily based around SQL it integrated well into our existing processes. SQL is a commonly used query language so resourcing the conversion work was achieved with existing staff with some additional on-line training from OHDSI and the European Health Data Evidence Network (EHDEN) Academy [18].

The OMOP clinical tables and the derived tables once connected to ATLAS were straightforward to work with. The pre-configured dashboards in ATLAS facilitated streamlined data visualisation. However, the real strength in ATLAS lies in the ability to rapidly construct concept sets, clinical cohorts, and design studies.

Another key advantage of the CDM, is its ability to facilitate network studies across multiple centres, both locally and across the globe. With ATLAS, research groups can design analysis packages and easily share them with other groups. These packages can then be imported and executed on local OMOP datasets. Such standardisation enables direct comparison of de-identified patient data between regions and countries without the need to transfer data from the source repository. This approach yields benefits in governance and security, allowing organisations to maintain control over data access while only allowing aggregated data to leave their systems. Additionally, from a security perspective, existing secure data repositories can be utilised for storing and analysing the data, eliminating the need to secure the data elsewhere.

One challenge we encountered, was the large amount of free text terms found in local EMR systems. We noted that the ‘*source of truth’* was with the text–where the most reliable and accurate information is found in the textual descriptions or notes that a GP reads, rather than in the numerical code values, such as SNOMED codes. In other words, when it comes to understanding patient conditions or information, the narrative or textual information is considered more authoritative and informative than the numerical codes. In some cases, textual descriptions did not match allocated codes and the codes were clearly erroneous. This made the task of mapping the terms time consuming with the potential to introduce errors. The ETL scripts to convert terms to the OMOP CDM can also be complex so we found it was important to document the scripts to ensure future maintainability.

A good understanding of data quality is central to the use of any dataset. It is especially important for OMOP datasets as the data is derived from source data and it has the potential to mask data quality issues, which only become apparent when comparing data to other datasets. During our quality assessment, we identified minor issues that required correction, such as discovering some values that were implausible. For instance, in some cases, missing dates of birth were recorded as 1900 in the EMR. This practice stems from the necessity for EMR systems to handle missing or incomplete data, including dates of birth, to uphold the accuracy and reliability of patient records. We also found whole tables that contained incomplete or no data, but this is normal with this type of primary care data. Two of the CDM tables were not populated in our data, the ‘PAYER_PLAN_PERIOD’ table. which refers to insurance data that is not applicable in the Australian context, and the ‘NOTE’ table as the narrative clinical note data is not extracted from the EMR source.

The data quality tool has a default threshold for incomplete data set at zero percent. This means any table or field with less than one-hundred percent data completion will be classified as a ’Fail.’ However, this default threshold was not suitable for our dataset. For instance, the ’CONDITION_OCCURRENCE’ table had only sixty-two percent of patients with an entry, which commonly occurs in this type of data due to reasons, such as GP documentation practices, where the condition occurrence maybe recorded as free text in the narrative notes. The recording of condition occurrence can also be influenced by factors related to clinical workflow, patient presentation, and limitations of the EMR system itself. Providentially, the data quality dashboard allows for customisation of the pass and fail thresholds to account for local conditions and prior knowledge, recognising that a one-size-fits-all approach may not be applicable in all cases.

The ETL proved to be a complex and time-consuming activity. But in future studies this could be made more efficient by modifying existing practise. The first and most obvious modification would be to have more coding in the source EMR systems rather than free text terms. This could be implemented as predicative text to reduce manual data entry for ‘time poor’ health care professionals. This would have the added benefit of allowing for validation of data input reducing typographical errors. However, changing proprietary systems is not a simple endeavour and will require cooperation from vendors and regulators.

In order to make the mapping process more manageable we employed a frequency-based approach to mapping terms. This relied on the fact that mapping frequently occurring terms converted a high percentage of required concepts. As an example, we covered 97% of medications by mapping only terms that appeared more than 200 times in our data. This is a pragmatic way of reducing the effort required to map terms. It is also important to note if rarely occurring concepts falling below the frequency threshold are to be studied, they can be mapped simply on a case-by-case basis. Hence, the frequency-based approach allows efficiency and flexibility in the mapping process.

To streamline the mapping process, we adopted a frequency-based strategy for term mapping, leveraging the observation that mapping commonly encountered terms effectively covered a significant portion of the necessary concepts. For instance, we achieved coverage for ninety-seven percent of medications by mapping terms that appeared in our data more than 200 times. This pragmatic approach serves to reduce the overall effort required for mapping while maintaining flexibility. It is worth noting that for rarely occurring concepts falling below the frequency threshold, they can still be mapped on a case-by-case basis when needed. In this manner, the frequency-based approach offers both efficiency and adaptability within the mapping process. The medication fields included, product names (generic and trade), strength, and pack size, we removed pack size to optimise RxNorm text matching in USAGI. Regarding medication vocabulary, Australia uses the Australian Medicines Terminology (AMT), however we chose to use RxNorm, because this is the standard drug vocabulary in the Observational Medical Outcomes Partnership-Common Data Model (OMOP-CDM). When dealing with situations where a one-to-one mapping of a RxNorm code to a medication is not possible, particularly with multi-ingredient medications (e.g., medications containing both pseudoephedrine and codeine), we employed RxNorm ingredient mapping. This approach allows for the application of multiple RxNorm codes to a single medication, ensuring accurate representation and comprehensive coverage of its constituent ingredients.

Another modification to the process that would help with subsequent primary care studies is to share the mappings produced for the ETL process. Indeed, we shared mappings with the University of New South Wales who had already mapped a number of general practice terms. However, in future shared mappings could potentially be shared programmatically via an Application Program Interface (API) with other research teams using Fast Healthcare Interoperability Resources (FHIR) servers, such as the Commonwealth Scientific and Industrial Research Organisation (CSIRO) Ontoserver [19]. This would streamline the process and cut down on manual tasks.

For the information contained in OMOP data sets to be used in research it is essential that good data governance is in place [12]. This ensures the rights of individual patients are respected and that the data is managed responsibly. Transparency in the governance process underpins trust in the data and is fundamental to successful research. We have developed an extensive data governance process that is being adopted by our data governance committee and we believe this provides a good model for other groups managing OMOP data to adopt and learn from.

In this research, we have made significant contributions to the ongoing research on the OMOP-CDM by validating it using real-world primary care data. Additionally, we have leveraged the data quality dashboard and discussed its utility within this paper. Our research also offers a comprehensive examination of implementing the open-source OMOP-CDM within a primary care data repository. By harnessing the PATRON primary care dataset, we illustrate the potential and wide-ranging implications of integrating the OMOP-CDM into real-world primary care settings. In doing so, we demonstrate the practicality and adaptability of adhering to the OHDSI-recommended conversion processes to achieve our research objectives.

### Future options for data linkage

As part of this program of work, we are also investigating patient record linkage between primary care and hospital datasets. Whilst this paper describes the conversion of a primary care data repository to the OMOP-CDM, we are also in the process of converting a hospital dataset to OMOP using the same linkage keys. This provides opportunity, as when linkage keys exist in both primary care and hospital data, records can be linked to create a more comprehensive patient record. This linkage method has previously been demonstrated by other groups [20–22]. In these studies, data from EMR’s have been enhanced with more detailed health data from other healthcare sources, such as cancer registries, to increase completeness of the datasets.

## Conclusion

The OMOP CDM’s widespread international use, support, and training provides a well-established pathway for data standardisation in collaborative research. Its compatibility allows the sharing of analysis packages across local and international research groups, which facilitates rapid and reproducible data comparisons. A suite of open-source tools, including the OHDSI Data Quality Dashboard, supports the model. Its simplicity and standards-based approach facilitates adoption and integration into existing data processes.

## Abbreviations

SQL: structured query language
OHDSI: Observational Health Data Sciences and Informatics
OMOP: Observational Medical Outcomes Partnership
EMR: Electronic Medical Record
Patron: Primary Care Audit, Teaching and Research Open Network
